The article "Noninvasive Evaluation of the Biomechanical Accommodations to Bolus Volume during Human Swallowing" was published in 2022. Journal: Appl Bionics Biomech.

# Noninvasive Evaluation of the Biomechanical Accommodations to Bolus Volume during Human Swallowing

**DOI:** 10.1155/2022/7146947

**Published:** 2022-10-14

**Authors:** Qiang Li, Kazuhiro Hori, Kazuhiro Murakami, Yoshitomo Minagi, Yoshinobu Maeda, Yongjin Chen, Takahiro Ono

**Affiliations:** ^1^State Key Laboratory of Military Stomatology & National Clinical Research Center for Oral Diseases & Shaanxi International Joint Research Center for Oral Diseases, Department of General Dentistry & Emergency, School of Stomatology, The Fourth Military Medical University, Xi'an, Shaanxi 710032, China; ^2^Department of Prosthodontics, Gerodontology and Oral Rehabilitation, Osaka University Graduate School of Dentistry, Suita 565-0871, Japan; ^3^Division of Comprehensive Prosthodontics, Niigata University Graduate School of Medical and Dental Sciences, Niigata 951-8514, Japan

## Abstract

Bolus volume is very important in the biomechanics of swallowing. By noninvasively characterizing swallow responses to volume challenges, we can gain more knowledge on swallowing and evaluate swallowing behavior easily. This study aimed to evaluate the impact of bolus volume on the biomechanical characteristics of oropharyngeal swallowing events with a noninvasive sensing system. Fifteen healthy male subjects were recruited and instructed to swallow 5, 10, and 15 ml of water. The sensing system consisted of a tongue pressure sensor sheet, bend sensor, surface electrodes, and a microphone. They were used to monitor tongue pressure, hyoid activity, surface EMG of swallowing-related muscles, and swallowing sound, respectively. In addition to the onset, the peak time and offset of the above four structures, certain characteristics, such as the duration, peak value, and interval of the structure motions, were measured during the different drinking tasks. The coordination between the hyoid movement and tongue pressure was also assessed. Although no sequence of the structural events changed with volume, most of the timings of the structural events were significantly delayed, except for certain hyoid activities. The swallowing volume did not affect the active durations of the monitored structures, the peak values, or intervals of tongue pressure and supra- and infrahyoid muscle activity, but certain hyoid kinetic phases were prolonged when a larger volume was swallowed. Additionally, sequential coordination between hyoid movement and tongue pressure was confirmed among the three volumes. These findings suggest that oropharyngeal structural movements change in response to bolus volume to facilitate safe swallowing. The noninvasive and quantitative measurements taken with the sensing system provide essential information for understanding normal oropharyngeal swallowing.

The article "Noninvasive Evaluation of the Biomechanical Accommodations to Bolus Volume during Human Swallowing" was published in 2022. Journal: Appl Bionics Biomech.

## 1. Introduction

Swallowing is one of the most basic and important physiological functions of human beings. This function involves many structural activities that naturally occur in a well-tuned rhythm simultaneously and sequentially [1]. As the size of the elderly population is growing rapidly worldwide, swallowing disorder is becoming increasingly prominent. Dentists are beginning to treat dysphagic patients more frequently than before. Therefore, dentists should fully understand oropharyngeal swallowing behaviors so that they can select optimal treatments.

Bolus volume is an important modulator of the biomechanical events that occur during oropharyngeal swallowing [2]. When boluses of different volumes are swallowed, volume accommodation occurs to guarantee safe and efficacious swallowing. While patients with neurologically impaired dysphagia may be at the risk of penetration and aspiration with large bolus volumes, small bolus volumes beyond a certain threshold may not trigger the automatic swallowing reflex [3]. Researchers have reported the effects of bolus volume on the tongue [4], hyoid [5], and swallowing-related muscles [6]. However, few studies have simultaneously monitored the effects of bolus volume on oropharyngeal structures with noninvasive methods.

Currently, videofluoroscopy (VF), which is considered as the gold standard, is commonly used to provide information on the movement of anatomic structures during swallowing. However, its drawbacks, especially its association with radiation exposure and time-consuming analysis, limit its widespread application. To overcome the weaknesses of VF and make the evaluation of swallowing convenient for patients and clinicians, various techniques have been explored [7]. Our group has established a sensing system composed of a tongue pressure sensor sheet, bend sensor, surface electrodes, and a microphone that can successfully and conveniently monitor the coordination among tongue pressure, swallowing-related muscle activities, and hyoid motion [8]. It is considered as a simple and noninvasive clinical method of evaluating the physiological and biomechanical aspects of oropharyngeal swallowing [8].

Hence, the primary objective of this study was to investigate and describe the impact of bolus volume on the sequence of oropharyngeal swallowing events noninvasively. The secondary objective of this study was to evaluate the dynamic characteristics of certain important structures related to bolus accommodation during swallowing. We hypothesized that in healthy individuals without dysphagia symptoms, these interrelationships would change with increasing volume in concert with normal motor modulation of the swallow mechanism.

The article "Noninvasive Evaluation of the Biomechanical Accommodations to Bolus Volume during Human Swallowing" was published in 2022. Journal: Appl Bionics Biomech.

## 2. Materials and Methods

### 2.1. Participants

Fifteen young healthy male participants (age range = 25–32 years) were enrolled in this study. All participants were in good health without severe malocclusion, symptoms or a history of swallowing difficulty, reflux symptoms, medications known to interfere with swallowing, speech disorders, structural disorders, cognitive disorders, or neurologic and/or muscular diseases. The study has been conducted in full accordance with the Declaration of Helsinki (1964). The Ethics Committee of Osaka University Graduate School of Dentistry reviewed and approved the study (No. H21-E32). All subjects provided informed consent.

### 2.2. Measuring Equipment

The measurement system used was a sensing system (Figure 1(a)) consisting of four noninvasive devices, that is, a tongue pressure sensor sheet (Figure 1(b)), surface electrodes (Figure 1(c)), a bend sensor (Figure 1(d)), and a microphone (Figure 1(e)). Tongue pressure was measured by the tongue pressure sensor sheet (100 Hz; thickness, 0.1 mm; measurement points Channel 1 to Channel 5 (Ch. 1–Ch. 5)) attached to the hard palate. Ch. 1–Ch. 3 were placed along the median line anteroposteriorly, and Ch. 4 and Ch. 5 were situated in the posterior–circumferential parts of the hard palate. The appropriately sized sensor sheet was selected from three sizes according to the participant's palate form [9, 10] and calibrated by applying negative pressure using a vacuum pump through an air duct; then, the sheet was attached to the hard palate with a sheet-type denture adhesive (Touch Correct II, Shionogi). Five surface electrodes (Duo-trode, Myotronics) were used to record the electromyography (EMG) signals of the suprahyoid muscle and infrahyoid muscle (SH EMG and IH EMG) [11, 12]. One pair of electrodes (*d* = 8 mm, interelectrode distance = 2 cm) was taped to the skin on the right side of the anterior belly of the digastric muscle. Another pair of electrodes were taped to the right side of the sternohyoid muscle. A single electrode was affixed to the forehead as the ground. The signals from the EMG electrodes were band-passed filtered (100 Hz–10 kHz), amplified (BA1104, Nihon Kohden), full-wave rectified and smoothed (time constant, 20 ms) using an application (MaP1038A, Nihon Santeku), and then, the signals were stored on a computer through an interface (PCI-3133A, Nihon Santeku) at a sampling rate of 10 kHz. To record the hyoid activity, the bend sensor (73.7 mm × 6.4 mm × 1.0 mm, 1000 Hz, MaP 1783BS1-056, Nihon Santeku), which was able to flexibly move with laryngeal motion, was taped on the skin along the midline of the frontal neck. Its tip was fixed at the level of the prominence of the thyroid cartilage when reaching the highest position during swallowing. The details of hyoid activity were mirrored noninvasively on the basis of the produced signal waveform [13]. Because the symmetry of the swallowing sound could be acquired bilaterally [14], a microphone (JM-0116, Ono-Sokki) was placed over the left lateral border of the trachea immediately inferior to the cricoid cartilage to detect the timing of the bolus passage through the entrance of esophagus [15].

The article "Noninvasive Evaluation of the Biomechanical Accommodations to Bolus Volume during Human Swallowing" was published in 2022. Journal: Appl Bionics Biomech.

### 2.3. Experimental Procedure

The participants included in this study were instructed to sit in an upright position with their heads supported by a headrest to avoid head retroflexion and to keep the Frankfort plane horizontal, with their feet touching the floor. Then, 5, 10, or 15 ml of water (37°C) was given to the participant during each trial, and the order of trials was randomized (http://www.researchrandomizer.org). The liquid was administered via a syringe, and the participant held the liquid on the mouth floor until they received a verbal command to swallow the entire volume at one time. The participant was asked to relax the tongue immediately after each trial. Three repetitions were performed for each bolus volume by each subject. The recorded tongue pressure and swallowing sound data were subsequently integrated on a personal computer through an interface board (PCD 100A, Kyowa Electric Instruments). The EMG data and the obtained signal from the bend sensor were amplified and stored on a personal computer through a separate interface board (PCI-3133A, Nihon Santeku). To ensure that all of the subjects felt comfortable and that all the devices worked properly, at least one successful performance was completed before the experimental data were recorded. To synchronize all the data, a trigger signal to start the measurement from the swallow scan was sent to the interface board (PCI-3133A, Nihon Santeku); then, the tongue pressure, EMG signals, hyoid motion, and swallowing sound were measured at the same time.

### 2.4. Data Analysis

Representative recordings of the tongue pressure, EMG signals of the swallowing-related muscles, hyoid movement, and swallowing sound with the sensing system are shown in Figures 1(f), 1(g), 1(h) and 1(i), respectively. The following parameters of the tongue pressure on each sensor were recorded: onset of tongue pressure (TP_on_), time of maximum tongue pressure (TP_max_), offset of tongue pressure (TP_off_), peak value of tongue pressure (TP_peak_), integrated area of tongue pressure, and duration of tongue pressure from TP_on_ to TP_off_ (Figure 1(f)). For the EMG of suprahyoid muscle (SH) and infrahyoid muscle (IH), the onset (EMG_on_), peak time (EMG_max_,), offset (EMG_off_), peak value (EMG_peak_), duration, and burst area were measured (Figure 1(g)). The onset time of each EMG burst was the time at which 2 standard deviations (SDs) were above baseline activity, and the offset time was the time at which 2 SDs were below baseline activity [16]. Additionally, certain time points on the laryngeal signal waveform produced by the bend sensor were used to represent the hyoid activity (Table 1), and certain hyoid active phases were defined in Table 2 [8, 10, 13]. With respect to the swallowing sound, because more than one spike was typically observed in the sound data, the spike with the largest amplitude was chosen as the reference time to compare the temporal sequence of biomechanical events during oropharyngeal swallowing (Figure 1(i)).

The article "Noninvasive Evaluation of the Biomechanical Accommodations to Bolus Volume during Human Swallowing" was published in 2022. Journal: Appl Bionics Biomech.

### 2.5. Statistical Analysis

All the data from 135 trials (15 subjects × 3 volumes × 3 trials) were analyzed with SPSS 17.0 software. To evaluate the sequential order of tongue pressure, muscle EMG activity, and hyoid activity, the uniformity of variance was first confirmed by the Kolmogorov–Smirnov test, and the significance of structural events was determined by repeated-measures analysis of variance (ANOVA) followed by the Bonferroni post hoc test. One-way ANOVA followed by the Bonferroni post hoc test was used to compare the durations of hyoid activity in each physiological phase, the parameters of tongue pressure at one site, the parameters of SH EMG, and the parameters of IH EMG. As for the significances of EMG parameters between SH and IH, the paired *t*-test was performed. The intraclass correlation coefficient was used to evaluate the correlations between T2 and TP_on_, T4 and TP_max_, as well as T5 and TP_off_ to assess the coordination between the hyoid motion and tongue activities. Statistical significance was set at *p* < 0.05. All the data were expressed as the mean ± SD.

## 3. Results

### 3.1. Volume Accommodation of the Temporal Sequence of Oropharyngeal Biomechanical Events

As shown in Figure 2, after the swallowing sound was set as the reference time, the sequence of events was timed clearly. When any volume of liquid was swallowed, the onset of hyoid slight movement (T1) occurred first, and then, the SH EMG_on_ and IH EMG_on_ occurred one after another. SH EMG_max_ and the onset of hyoid rapid movement (T2) occurred simultaneously, followed by IH EMG_max._ Meanwhile, TP_on_ occurred along the midline of the hard palate from the front to the back (Ch. 1–Ch. 3), with the signals from Ch. 4 and Ch. 5 arising at the palatal circumferential part. TP_max_ at each site occurred earlier than the onset of the stationary phase of the hyoid (T4). When the hyoid began to descend (T5), SH EMG_off_, IH EMG_off_, and TP_off_ at each site disappeared at nearly the same time.

The article "Noninvasive Evaluation of the Biomechanical Accommodations to Bolus Volume during Human Swallowing" was published in 2022. Journal: Appl Bionics Biomech.

The overall sequence of events did not differ across the three volumes. However, we observed that an increasing bolus volume obviously delayed the onset and termination of most of the structural events, with significant differences for TP_on_ at each site between volumes of 5 and 15 ml (all *p* < 0.05), TP_max_ at Chs. 3–5 between volumes of 5 and 15 ml (all *p* < 0.05), and TP_on_ at Ch. 4 and Ch. 5 between volumes of 5 and 10 ml (both *p* < 0.05). In addition, the offset of the stationary phase of the hyoid (T5) and the offset of hyoid movement (T6) occurred later for a volume of 15 ml than for a volume of 5 ml (both *p* < 0.05). Only the onset of hyoid rapid movement (T2), onset of the stationary phase of the hyoid (T4), and SH EMG_max_ occurred slightly earlier as the bolus volume increased, with significant differences of T2 and SH EMG_max_ between volumes of 5 and 15 ml (both *p* < 0.05).

### 3.2. Tongue Pressure Characteristics Related to Bolus Volume Accommodation

The duration of tongue pressure at each site did not vary with the swallowing volume (*p* > 0.05, Figure 3(a)). Additionally, no significant volume dependence was found for TP_peak_ (*p* > 0.05, Figure 3(b)) or integrated area of tongue pressure (*p* > 0.05, Figure 3(c)).

### 3.3. Swallowing-Related Muscle Characteristics Related to Bolus Volume Accommodation

As shown in Figure 4, the durations, peak values, and EMG burst area of the suprahyoid muscle were similar across the three volumes (*p* > 0.05). Similar results were found in the infrahyoid muscle (*p* > 0.05). Additionally, no significances between suprahyoid muscle and infrahyoid muscle were noted for the above-tested characteristics (*p* > 0.05).

### 3.4. Hyoid Characteristics Related to Bolus Volume Accommodation

As shown in Figure 5, as the swallowing volume increases, there was a decreasing trend in the duration of the hyoid slight motion phase (T1–T2) and an increasing trend in the durations of the hyoid elevation phase (T2–T4), hyoid stabilization phase (T4–T5), and hyoid active phase (T2–T5). Significant volume-dependent tendencies for T4–T5 and T2–T5 were confirmed between the volumes of 10 and 15 ml (both *p* < 0.05) as well as between the volumes of 5 and 15 ml (both *p* < 0.05). No obvious volume effects were found for the duration of the hyoid descent phase (T5–T6) or duration of the hyoid motion phase (T1–T6) (*p* > 0.05).

### 3.5. Volume Effects on the Coordination between Hyoid Movement and Tongue Pressure

The correlations between time points on the hyoid signal waveform and tongue pressure were shown in Table 3. Significant positive correlations were found between T2 and TP_on_s at Chs.1–5 with a low-to-moderate correlation coefficient during swallowing either volume (all *p* < 0.05) except for TP_on_ at Ch. 3 when swallowing 15 ml (*p* > 0.05). In addition, T4 had positive associations with TP_max_s at Chs.1–5 with a moderate correlation coefficient (all *p* < 0.05). Moreover, there were significant positive correlations between T5 and TP_off_s at all Chs. with a moderate-to-high correlation coefficient (all *p* < 0.05).

The article "Noninvasive Evaluation of the Biomechanical Accommodations to Bolus Volume during Human Swallowing" was published in 2022. Journal: Appl Bionics Biomech.

## 4. Discussion

To our knowledge, this is the first study to successfully and noninvasively evaluate the biomechanical accommodations to bolus volume during human oropharyngeal swallowing with a sensing system, that is, a sensor sheet measuring tongue pressure, a bend sensor measuring hyoid motion, electrodes measuring muscle EMG signals, and a microphone measuring the timing of bolus passage through the entrance of the esophagus.

We found that the temporal order of events did not differ by bolus volume when the subjects swallowed three different volumes of water. The increased volume only delayed the structural onset, peak, and offset time. These findings are consistent with the conclusion from a kinematic analysis using 320-row area detector CT [7], in which the events related to many oropharyngeal structures (such as the tongue, hyoid, and upper esophageal sphincter (UES)) remained stable during swallowing of 3–20 ml. Our results and those of a previous study suggested that the event sequence during healthy oropharyngeal swallowing is not affected by bolus volume. Meanwhile, the sensibility of the used sensing system could be reflected based on the present results.

After comparing certain hyoid activities, we noticed significant differences in certain hyoid events, that is, T2, and T5, during swallowing between the volumes of 5 and 15 ml. T2 represents the onset of rapid movement of the hyoid toward the highest position along the anterosuperior direction [13]. We posited that an earlier occurrence of T2 during the swallowing of 15 ml of water is a biomechanical preparation of the hyoid for the upcoming large volume of liquid. Hoffman et al. [17] considered earlier hyoid excursion subsequent to a larger bolus volume may be an accommodation to a lower hyoid resting position to maintain the integrity of swallowing. Physiologically, a larger bolus volume results in a longer bolus length in the mouth and pharynx [18]. Correspondingly, it is mandatory for the hyoid to remain at the highest position for a longer stabilization time and descend later to facilitate the passage of a larger bolus. As a result of the earlier appearance of T2 and later appearance of T5, the major effect of bolus volume was that the hyoid slight motion phase (T1–T2) shortened and the hyoid stabilization phase (T4–T5) and the hyoid active phase (T2–T5) lengthened as the volume increased. However, the data of this study failed to show significant differences in the hyoid total motion phase (T1–T6) as a function of volume for liquids ranging from 5 to 15 ml in the target volume. Many studies [7, 19, 20] have also reported that the hyoid burst duration does not obviously differ by bolus volume, although the hyoid velocity and excursion distance are affected by the volume.

The article "Noninvasive Evaluation of the Biomechanical Accommodations to Bolus Volume during Human Swallowing" was published in 2022. Journal: Appl Bionics Biomech.

For tongue pressure, we identified significant differences in the onset of the tongue pressure at each channel and the peak time of the tongue pressure in posterior parts. Because the mouth floor should prepare to hold more volume when larger volumes are swallowed, the tongue needs to raise its initial position. Then, the tongue tip needs to scoop up the water from its initial higher position and rise to contact the hard palate and then the other parts of the tongue when the individual receives a swallowing command. This action will take more time when a larger volume compared with a smaller volume is swallowed. Therefore, it is reasonable that TP_on_ was delayed at the sites of the anterior and posterior–circumferential parts of the hard palate (Ch. 1, 4, and 5) for a volume of 15 ml compared with that of a volume of 5 ml. In this study, TP_max_ was delayed only for Ch. 3–5. We consider that the peak tongue pressure at posterior parts of the hard palate occurred later due to precise central nervous regulation to maintain the hyoid at its most anterosuperior position, thereby facilitating UES opening and epiglottis closure for safe swallowing. In fact, the correlations between T4 and TP_max_ strengthened as the swallowing volume increased, indicating that the tongue pressure adapted to the bolus volume during oropharyngeal swallowing. Additionally, TP_off_ at each site became delayed as the swallowing volume increased, but the differences did not reach significance in the present study. Similar findings were also reported by Yano et al. [21], who reported that the onset time, peak time, and offset time of tongue pressure along the midline during the swallowing of 5 ml of liquid preceded those during the swallowing of 15 ml of liquid. Concerning the tongue pressure-related parameters, that is, duration, peak value, and integral value, there were no obvious volume-dependent tendencies in the current study.

The article "Noninvasive Evaluation of the Biomechanical Accommodations to Bolus Volume during Human Swallowing" was published in 2022. Journal: Appl Bionics Biomech.

Cock et al. [22] recorded intramuscular surface submental EMG (SM-EMG) signals in eight healthy volunteers while they swallowed 0.9% saline boluses of 2, 5, 10, and 20 ml. The researchers found that the temporal sequence of SM-EMG events gradually moves backward as the volume increases. Except for the similar findings of delayed onset and offset time, we noted an earlier occurrence of SH EMG_max_ when swallowing 15 ml water compared with 5 ml water. This discrepancy might be the result of different electromyography techniques being used. As the suprahyoid muscle plays an important role in elevating the hyoid toward the highest position [23], the fact that the peak time of the suprahyoid muscle matches the onset of rapid movement of the hyoid well is considered logical. In the above research, the SM-EMG duration did not change with the testing volume. Dantas et al. also showed that bolus volume (2–20 ml) did not change the timing or duration of SM-EMG or IH EMG activity [24]. However, one study [25] in 14 normal subjects showed opposite results of a statistically longer duration of SM-EMG activity as the swallowing volume increased from a dry condition to 20 ml water. Our data confirm that the duration, peak value, and burst area of the swallowing-related muscle EMG signals did not significantly change with the swallowing volume. Generally, the natural and free-drinking sip volume for healthy volunteers is approximately 24 ml [26]. Based on the volumes of 5–15 ml liquid swallowed in this study, we consider that swallowing volumes less than the natural swallowing size have no effects on the hyoid total motion phase (T1–T6) or the tongue pressure or EMG parameters. However, whether the changes occur when the swallowing volume is larger needs to be studied further.

Previous studies have confirmed the prolonged duration of tongue pressure and time to peak pressure as well as reduced pressure gradient in the dysphagic aged group [27]. Age-related alterations of EMG activities are also evident in the supra- and infrahyoid muscles [28, 29]. Additionally, reduced displacement and velocity of the hyoid bone during swallowing are obvious in aging dysphagic patients [30, 31]. Therefore, we consider that any abnormalities of tongue pressure, surface EMG of swallowing-related muscles, hyoid activity, or their biomechanical accommodations to bolus volume in the elderly during swallowing could serve as potential clinical indicators to reflect dysphagic condition.

While some phenomena and several significant differences were observed between the volumes of 5, 10, and 15 ml during the swallowing of water, there were still limitations to this study. First, the sample size was relatively small. Second, most of the participants involved in this study were young adults. Additional research should be conducted in different age groups to obtain a systematic and comprehensive conclusion, given that age is known to impact temporal measures of swallowing [32, 33]. Third, all the participants in this investigation were normal individuals. Sensing measurements from individuals with swallowing disorders may reveal results different from those observed in the present study. All of the above limitations should be taken into consideration in the future.

The article "Noninvasive Evaluation of the Biomechanical Accommodations to Bolus Volume during Human Swallowing" was published in 2022. Journal: Appl Bionics Biomech.

## 5. Conclusions

In conclusion, the order of the structural events did not vary with changing fluid volume, but most of the structural events were delayed, except for hyoid anterosuperior excursion. The larger volume prolonged the duration of the hyoid being at its highest position and the hyoid active phase, although no obvious effects of volume on the tongue pressure or swallowing-related muscle EMG signals were confirmed. Our results demonstrate that the close correlation between hyoid activity and tongue pressure remained stable regardless of the liquid volume. These findings may not only enable us to determine the biomechanical accommodations to bolus volume that occur during human oropharyngeal swallowing but also provide us a simple and noninvasive method to evaluate the physiology of deglutition in healthy individuals as well as patients with dysphagia at the dental chairside and bedside clinically.

## Figures and Tables

**Figure 1:** Schematic representations of the sensing system and recordings. (a) A subject with tongue pressure sensor sheets, surface electrodes, bend sensors, and microphones. (b) Tongue pressure sensor sheet. (c) Surface electrodes. (d) Bend sensor. (e) Microphone. (f) The tongue pressure waveform. (g) The EMG of swallowing-related muscle. (h) The laryngeal signal waveform and marked time point. (i) The swallowing sound waveform. TP_on_, onset of tongue pressure; TP_max_, time of maximum tongue pressure; TP_off_, offset of tongue pressure; TP_peak_, peak value of tongue pressure; EMG_on_, onset of electromyography; EMG_max_, time of peak electromyography, EMG_off_, offset of electromyography; EMG_peak_, peak value of electromyography; T1, onset of hyoid slight movement; T2, onset of hyoid rapid movement; T4, onset of stationary phase of the hyoid; T5, offset of the stationary phase of the hyoid; T6, offset of hyoid movement. T3 and T7 were confirmed to be meaningless for hyoid activity.

**Figure 2:** Temporal sequence of biomechanical events during oropharyngeal swallowing. The red line notes the swallowing sound as the reference time. T1, onset of hyoid slight movement; T2, onset of hyoid rapid movement; T4, onset of stationary phase of the hyoid; T5, offset of stationary phase of the hyoid; T6, offset of hyoid movement. T3 and T7 were confirmed to be meaningless for hyoid activity; Ch. 1–Ch. 5, Channel 1 to Channel 5.

The article "Noninvasive Evaluation of the Biomechanical Accommodations to Bolus Volume during Human Swallowing" was published in 2022. Journal: Appl Bionics Biomech.

**Figure 3:** Effects of bolus volume on tongue pressure parameters. (a), Duration of tongue pressure. (b), Magnitude of tongue pressure. (c), Integrated area of tongue pressure. Ch. 1–Ch. 5, Channel 1 to Channel 5. Data were expressed as the mean ± standard deviation (SD).

**Figure 4:** Effects of bolus volume on swallowing-related muscles parameters. (a) Duration of swallowing-related muscle. (b) Peak value of swallowing-related muscle. (c) EMG burst area of swallowing-related muscle. Data were expressed as the mean ± standard deviation (SD).

**Figure 5:** Effects of bolus volume on hyoid active phases. T1–T2, hyoid slight motion phase; T2–T4, hyoid elevation phase; T4–T5, hyoid stabilization phase at the most anterior-superior position; T5–T6, hyoid descent phase; T2–T5, hyoid active phase; T1–T6. hyoid total motion phase. Data were expressed as the mean ± standard deviation (SD). ∗*P* < 0.05.

**Table 1:** Definitions of time points on the laryngeal signal waveform recorded by the bend sensor.

Time point	Synchronized indication for hyoid motion
T1	Onset of hyoid slight movement
T2	Onset of hyoid rapid movement
T3	None
T4	Onset of stationary phase of the hyoid
T5	Offset of stationary phase of the hyoid
T6	Offset of hyoid movement
T7	None

**Table 2:** Definitions of phases on the laryngeal signal waveform recorded by the bend sensor.

Phase	Definition	Synchronized indication for hyoid motion
Preliminary phase of waveform	T1–T2	Hyoid slight motion phase
Former part of the downward phase of waveform	T2–T4	Hyoid elevation phase
Latter part of the downward phase of waveform	T4–T5	Hyoid stabilization phase at the most anterior-superior position
Recovery phase of waveform	T5–T6	Hyoid descent phase
Downward phase of waveform	T2–T5	Hyoid active phase
Total phase of waveform	T1–T6	Hyoid total motion phase

**Table 3:** Correlation coefficient between hyoid movement and tongue pressure among different volumes.

Time points on the laryngeal waveform	Event on the tongue pressure	*r* (*p*)		
		5 ml	10 ml	15 ml
**T2**	**Ch. 1 TP**_**on**_	0.329 (***0.045***)	0.331 (***0.047***)	0.520 (***0.001***)
	**Ch. 2 TP**_**on**_	0.361 (***0.020***)	0.361 (***0.021***)	0.377 (***0.024***)
	**Ch. 3 TP**_**on**_	0.674 (<***0.001***)	0.589 (<***0.001***)	0.139 (0.406)
	**Ch. 4 TP**_**on**_	0.415 (***0.039***)	0.489 (***0.002***)	0.420 (***0.037***)
	**Ch. 5 TP**_**on**_	0.344 (***0.022***)	0.462 (***0.002***)	0.430 (***0.006***)
**T4**	**Ch. 1 TP**_**max**_	0.497 (***0.004***)	0.608 (<***0.001***)	0.619 (<***0.001***)
	**Ch. 2 TP**_**max**_	0.455 (***0.008***)	0.426 (***0.006***)	0.577 (<***0.001***)
	**Ch. 3 TP**_**max**_	0.482 (***0.003***)	0.541 (<***0.001***)	0.559 (<***0.001***)
	**Ch. 4 TP**_**max**_	0.436 (***0.008***)	0.628 (<***0.001***)	0.643 (<***0.001***)
	**Ch. 5 TP**_**max**_	0.466 (***0.006***)	0.461 (***0.003***)	0.470 (***0.003***)
**T5**	**Ch. 1 TP**_**off**_	0.748 (<***0.001***)	0.805 (<***0.001***)	0.544 (<***0.001***)
	**Ch. 2 TP**_**off**_	0.658 (<***0.001***)	0.613 (<***0.001***)	0.548 (<***0.001***)
	**Ch. 3 TP**_**off**_	0.701 (<***0.001***)	0.656 (<***0.001***)	0.657 (<***0.001***)
	**Ch. 4 TP**_**off**_	0.777 (<***0.001***)	0.715 (<***0.001***)	0.563 (<***0.001***)
	**Ch. 5 TP**_**off**_	0.625 (<***0.001***)	0.727 (<***0.001***)	0.562 (<***0.001***)

Values are given as *r* (*p*). Ch., channel. TPo_n_, onset of tongue pressure; TP_max_, time of maximum tongue pressure, TP_off_, offset of tongue pressure; T2, onset of hyoid rapid movement; T4, onset of stationary phase of the hyoid; T5, offset of stationary phase of the hyoid. Values shown in bold text in the bracket are statistically significant.

The article "Noninvasive Evaluation of the Biomechanical Accommodations to Bolus Volume during Human Swallowing" was published in 2022. Journal: Appl Bionics Biomech.

## Data Availability

The datasets used and analyzed during the current study are available from the corresponding author upon reasonable request.
